This article has been retracted.

# Formation of recombinant bifunctional fusion protein: A newer approach to combine the activities of two enzymes in a single protein

**DOI:** 10.1371/journal.pone.0265969

**Published:** 2022-04-01

**Authors:** Patel Nilpa, Kapadia Chintan, R. Z. Sayyed, Hesham El Enshasy, Hala El Adawi, Alaa Alhazmi, Atiah H. Almalki, Shafiul Haque

**Affiliations:** 1 Department of Plant Molecular Biology and Biotechnology, ASPEE College of Horticulture and Forestry, Navsari Agricultural University, Navsari, Gujarat, India; 2 Department of Microbiology, PSGVP Mandal’s S. I. Patil Arts, G B Patel Science & STKVS Commerce College, Shahada, Maharashtra, India; 3 Department of Entomology, Asian PGPR Society for Sustainable Agriculture, Auburn University, Auburn, AL, United States of America; 4 Institute of Bioproduct Development (IBD), Universiti Teknologi Malaysia (UTM), Skudai, Johor Bahru, Malaysia; 5 School of Chemical and Energy Engineering, Faculty of Engineering, Universiti Teknologi Malaysia (UTM), Skudai, Johor Bahru, Malaysia; 6 City of Scientific Research and Technology Applications (SRTA), New Burg Al Arab, Alexandria, Egypt; 7 Medical Laboratory Technology Department, Jazan University, Jazan, Saudi Arabia; 8 SMIRES for Consultation in Specialized Medical Laboratories, Jazan University, Jazan, Saudi Arabia; 9 Department of Pharmaceutical Chemistry, College of Pharmacy, Taif University, Taif, Saudi Arabia; 10 Addiction and Neuroscience Research Unit, College of Pharmacy, Taif University, Al-Hawiah, Taif, Saudi Arabia; 11 Research and Scientific Studies Unit, College of Nursing and Allied Health Sciences, Jazan University, Jazan, Saudi Arabia; 12 Bursa Uludağ University Faculty of Medicine, Görükle Campus, Nilüfer,Bursa, Turkey; Mendel University of Agriculture and Forestry: Mendelova univerzita v Brne, CZECH REPUBLIC

## Abstract

The tissue of insects, pests, and fungi has a chitin layer followed by protein in the cell membrane. The complete biodegradation of chitin and protein-present in the waste requires the action of two enzymes, namely chitinase, and protease. Combining chitinase and protease in a single protein/enzyme will serve as a bifunctional enzyme that can efficiently degrade the chitin and protein-rich biomass. The present study was aimed to fuse these two enzymes to produce a single protein and study the kinetics of the recombinant fusion protein. A chitinase and alkaline protease genes were isolated, cloned, and expressed successfully as a fusion product in heterologous host *Escherichia coli*. The two native genes were successfully fused in *E*.*coli* by using flexible glycine–serine (G_4_S)_2_ linker (GGGGS, GS linker). The recombinant fusion protein in *E*.*coli* showed hydrolyzed chitin and protein on chitin and bovine serum albumin agar plates confirming the successful cloning and expression of chitinase and protease enzymes in a single fusion protein. The common pUC18-T7 mini vector with the ompA signal sequence helps the extracellular expression of fusion protein efficiently. The native gel electrophoresis revealed a molecular mass of purified protein as 92.0 kDa. The fusion protein’s maximal chitinase and protease activity occurred at pH 5.0 and 8.0 and 30 ^0^C, respectively resembling the individual enzymes’. In the kinetic studies of the fusion protein, it was observed that the presence of metal ions such as Cu^2+^, Na^2+^, and Ca^2+^; significantly enhanced the enzyme activities while organic solvents oxidants and chemicals have drastically affected the activities of both the enzymes in the fusion protein. No such fusion protein has been produced in a heterologous host yet. The reports on fusion protein with biomass-degrading capacity are also scarce. This is probably the first report of a bifunctional chitinase/protease expressed in *E*. *coli*.

## Introduction

Chitin is the most abundant, water-insoluble homopolymer of N-acetyl D-glucosamine (GlcNAc) just next to cellulose and lignin [1]. It is present in most invertebrates, the cuticle of nematodes, the cell wall of filamentous fungi, and the cuticle of arthropods [2]. Chitin, being a natural product, is continuously synthesized and degraded in the natural environment through chitinase. Chitinases (EC 3.2.1.14) are hydrolytic enzymes that cleave glycosidic bonds of chitin to produce GlcNAc and N-acetyl chitooligosaccharides (COSs) [3, 4]. Chitinase has received much commercial attention recently due to the increased demand for its reaction products such as GlcNAc and COSs in food industries and ethanol production and its application as a biocontrol agent against phytopathogenic fungi [5, 6]. Various microorganisms secrete different families of chitinases [7, 8], however, bacterial chitinase is the best source of chitinase, as it is easily regulated, its production is easily scaled up, it is produced extracellularly and in large quantities in shorter time. The microbes produce multiple chitinases for the complete degradation of chitin into monomers. Bacterial chitinase gradually cleaves chitin and probably generates a better end product than individual enzymes [9]. The use of cloned bacterial chitinase has been reported in a few bacterial genera [3, 10–19].

Proteases (E.C.3.4.21) are the hydrolytic enzymes that cleave peptide bonds and thus release amino acids and /or short-chain oligopeptides. Proteases have become industrially significant enzymes, acquiring about 60% share of the global enzyme market, accounting for about $ 2.21 billion in value. They are widely used in agriculture, pharmaceuticals, food processing, detergent, leather processing, etc. [20, 21]. Proteases have been produced by plants, animals, fungi, and bacteria [22–24]. However, microbial protease is preferred over plant or animal sources due to their higher activity ease in genetic modification, ample availability, convenient processing, and safe and cost-effective production, besides high stability and ability to function over the broader pH and temperature range [25]. Cloning the protease gene and its expression in *E*. *coli* has been reported in a few bacterial genera [26–32]. Among the different bacterial sp. *Bacillus* sp. has been more frequently studied and used to synthesize diverse and industrially important protease, as it produces the enzymes extracellularly, thus offers ease in the extraction and recovery, and the fermentation process is conveniently regulated [33].

Enzymes from wild strains have a narrow range of working temperature and pH, less stability, and more sensitivity to metal ions, solvents, detergents, oxidants, feed-back inhibitions, etc. Gene cloning of commercially important enzymes in the fast-growing host that also gives better expression, easy recovery and purification, higher enzyme yield, and aid into the desired features to the enzyme has been the goal of making industrially valuable enzymes.

The co-expression strategies have the limitation of low transformation efficiency and inconvenient screening during co-expression. Constructing a bifunctional/trifunctional gene could be an effective approach [34–39].

Although there are reports on the cloning of Chitinases and proteases; there are no reports on the cloning of two individual enzymes to produce a single fusion protein that possesses chitinase and protease activities. Thus, there is a need to produce a single fusion protein that exhibits two enzymes useful in the biodegradation of chitin and protein-rich wastes. The present study aimed at cloning, expression, and biochemical characterization of a single fusion gene product so that a single protein will have multifunctional activities.

## Materials and methods

### Bacterial strains, vector, chemical reagents, and culture conditions

The *Bacillus circulans* strain MTCC 7906 (Accession No.JN645176.1) for alkaline protease and *Serratia marcescens* strain GPS5 (Accession No.KX579968.1) for chitinase D and *E*. *coli* BL21 (DE3); an expression host was cultured overnight in LB broth at 30°C. These bacterial cultures and the extracellular expression vector pUC18T-mini-Tn7T-Tp-gfpmut3 were procured from the SLS research Pvt. Ltd. India. 5-Bromo-4-chloro-indolyl-β—galactopyranoside (X-Gal), isopropyl thiogalactoside (IPTG), and antibiotics (ampicillin and gentamycin) were procured from Merck (Germany) and used for the selection of transformed clones. All other chemical reagents were purchased from SLS Research Pvt. Ltd., India

#### Cloning of chitinase and protease genes

The genomic DNA of B.circulans strain MTCC 7906 and S.marcescens GPS5 was isolated from the overnight grown cultures of these organisms [40], and purity of the separated DNA was confirmed by agarose gel electrophoresis.

PCR amplified the gene encoding chitinase and protease from genomic DNA with the primers mentioned in Table 1. The laboratory designed these primers to remove a deduced signal sequence so that protein can be targeted to the extracellular site using the ompA signal sequence [41]. The rrnB transcription termination sequence was used to termination the transcription process. The amplified fragments were checked on the agarose gel electrophoresis for their expected band size. The sense and antisense strands of the linker (GGGGSGGGGS) were annealed by placing 10 ng each in PCR tubes and incubated under a PCR machine with a touchdown cycle from 95°C to 25°C with a gradual decrease of 5°C for every 5 min and incubated further at 25°C. The chitinase gene amplicon, protease gene amplicon, and linker were added to the PCR mixture. The overlapping primer was used to amplify the entire sequence as a long consensus [42] (Table 1). The amplified PCR products were analyzed through 1.5% agarose gel electrophoresis prepared in 1x TBE buffer and run for 20 min. at 7V/cm. The size of the amplified DNA fragments was determined on agarose gel by comparing with the 100+500 bp DNA ladder and photographed under the Bio-Rad Gel documentation system. Three constructs, namely (i) protease, (ii) chitinase, and (iii) chitinase fused with protease, were constructed by using flexible glycine–serine peptide linker (GGGGS, (G4S)2) [43]. The amplified and purified fragments were inserted into the vector pUC18 mini-Tn7T purchased from add gene, USA. The fusion sequence was treated with KpnI (GGTACC) restriction enzyme to create 3’overhang. The BamHI site (GGATCC), lac UV5 promoter, shine-Dalgarno sequence, ompA (Signal Sequence for secretion), and spacer sequences were synthesized as a separate unit (Table 1; sequence No. 10). The regulatory sequence along with BamHI at the 5’ end was ligated with the fusion product. The same sequence was treated with the mentioned restriction enzyme to create a 5’ cohesive end and mixed with the linear vector pUC18miniTn7 in the ratio of 1:5 (Vector: Insert) (Fig 1).

**Fig 1:** The map of pUC18-T7 mini vector with *E*.*Coli* rrnB transcription termination. Lac promoter (Blue color), Lac UV 5 Promoter (Blue color), Lac Operator (Blue color), Fusion Gene (purple color), rrnB T1 terminator (Color less), Ampicillin Resistant gene AmpR and pMB1 origin of replication.

**Table 1:** The list of the primers used in the present study.

Primer	Nucleotide sequence
FPChi	5’- ATG GCC TAT CTC TCC GTC GGC T -3’
RPChi	5’- GGTACCTTAATGGTGATGGTGATGGTGCCG TTT CTC GCC TTT TAT GTT CAG CGA -3’ (KpnI RE) (Stop) (HIS TAG)
FPP	5’- ATG GTT GGG TAC TCT ATG GTA CAA ATG GTG A -3’
RPP	5’- CAG AAA ATT CCG TTC CCG GCC AA -3’
RPP with overhang	5’- GGTACCTTAATGGTGATGGTGATGGTGCAG AAA ATT CCG TTC CCG GCC AA -3’ (KpnI RE) (Stop) (HIS TAG)
Linker sequence	5’GGCGGCGGCGGCAGCGGCGGCGGCGGCAGC-3’
Complementary Linker sequence	5’-GCTGCCGCCGCCGCCGCTGCCGCCGCCGCC-3’
FPP	5’GCGGCGGCGGCAGCGGCGGCGGCGGCAGCATGGTTGGGTACTCTATGGT-3’ **Overhang at 5’ end of Protease gene**
RPChi	5’-CTGCCGCCGCCGCCCCGTTTCTCGCCT-3’ **Overhang to the 5’ Protease gene**
BamHI -M10K10 lacuv5-promoter -SD-ompA-Spacer	5’GGATCCTCACTCATTAGGCACCCCAGGCTTTACACTTTATGCTTCCGGCTCGTATAATGTGTGGAATTGTGAGCGGATAACAATTTCACACAGGAAACAGCTAGGAGGATGGAAACCCTGTATAGCCTGTATAGCACCCATCGCGCGCTGGCGATTCTGGAAGCGCTGGCGATTCTGGAAGCGCTGGCGGTGGCGCTGGCGCTGGCGCTGGAAGCGCTGGCGGGCCTGTATCCGCATGAAGCGCTGGCGACCCATCGCGTGGCGCTGGCGCTGGCGGGCATTAACGCGCTGGCGGGCGGCGGCGGCAGCGGCGGCGGCGGCAGC-3’

*FPC:- Forward primer for cellulase, RPC:- Reverse primer for cellulase, FPChi:- Forward primer for chitinase, RPChi:- Reverse primer for chitinase, FPP:- Forward primer for protease, RPP:- Reverse primer for protease, SD:- Shine-Dalgarno sequence, ompA:- Signal sequence for *E*. *coli*.

The chemically competent *E*. *coli* BL21 (DE3) were mixed with the recombinant plasmids and transformed using the heat shock method [44]. The transformants were grown on an LB plate containing ampicillin and gentamycin (100 μg/mL each) at 30°C for 24 h and observed for the appearance of growth of transformants. The transformed cells were then picked from the plates and incubated in the antibiotic-containing LB broth at 30°C for 24 h and used for further study.

### Estimation of enzyme activities of the different constructs

Estimation of chitinase and protease activity was performed on basal agar plates containing (g/L) K_2_HPO_4_; 0.3, KH_2_PO_4_; 0.7_,_ MgSO_4_; 0.5, FeSO_4_; 0.01, MnCl_2_; 0.001, ZnSO_4_; 0.001, and yeast extract; 5.0 separately amended with 1% azo-casein and 1% colloidal chitin. The transformed cells having fusion protein were grown on these plates at 30°C for 72 h. Following the incubation, the chitin agar plate was stained with 0.1% congo red and observed for the zone of chitin hydrolysis. Azocasein plate was observed for the zone of casein (protein) hydrolysis around the bacterial colonies.

### Induction and purification of enzymes

*E*. *coli* BL21 (DE3) transformed with the corresponding expression vector was grown overnight at 30°C in LB supplemented with antibiotics. The next day, 100 μL of each culture broth was inoculated in 10 mL of fresh LB medium supplemented with antibiotics (ampicillin and gentamycin @100 μg/mL) and incubated at 30°C for 45 min., followed by the addition of 400 μM/mL of IPTG and further incubation at 30°C for 2 h to get 10^8^ numbers of cells/mL of culture. The one mL of each culture was transferred to their respective substrates containing LB broth. The induction of enzymes was carried out by providing 200 μM/mL IPTG, and then the cells were allowed to grow further at 30°C for 72 h. The broths were centrifuged at 10,000 rpm for 10 min. and the supernatants were dialyzed against Tris buffer (pH 7.5) to remove media ingredients. Enzymes were purified using Ni-Nitrilotriacetic acid agarose column for His tagged dialyzed proteins (Takara Bio Inc., USA). The columns were equilibrated with equilibration buffer (50 mM sodium phosphate, 300 mM sodium chloride, 20 mM imidazole; pH 7.4) followed by washing with His60 Ni wash buffer (50 mM sodium phosphate, 300 mM sodium chloride, 40 mM imidazole; pH 7.4) and incubated at 30°C for 5–7 min. To this tube, 10–20 mL of dialyzed clear protein was added and eluted with 15 mL elution buffer (50 mM sodium phosphate, 300 mM sodium chloride, 300 mM imidazole; pH 7.4). The eluted proteins were collected and assayed for chitinase and protease activities.

#### Chitinase assay

Chitinase activity was estimated according to the method of Lee et al. [45]. The reaction mixture consisting of different volumes of enzyme solution (60 μL, 300 μL, and 500 μL for crude, dialyzed, and purified respectively) and 4 mL (1% w/v) of colloidal chitin (prepared from shrimp shells in 100 mM sodium acetate buffer (pH 5.5) was incubated at 30°C for 60 min. The reducing sugars were estimated analyze by the Somogyi–Nelson method [46], using GlcNAc as the standard. One unit (U) of chitinase activity was defined as the amount of enzyme that liberated one μM of GlcNAc per minute per mL under the assay conditions. According to Lowry et al. [47], the amount of available proteins was measured, using bovine serum albumin (100–1000 μg/mL) as the standard.

#### Protease assay

Protease activity was measured according to the method of Aretz et al. [48]. The reaction mixture consisting of different volumes of enzyme solution (60 μL, 300 μL, and 500 μL for crude, dialyzed, and purified respectively), 5 mL substrate (1% casein) was incubated at 30°C for 10 min and followed by adding 5 mL of 100 mM Trichloroacetic acid (TCA) and mixed thoroughly. The solutions were filtered through Whatman filter paper and checked for color development due to the release of tyrosine. The amount of tyrosine from the filtrate was measured according to the Lowry method [47], and the amount of tyrosine was calculated from the standard curve of tyrosine (100–1000 μg/mL). One unit of protease was defined as the amount of enzyme that liberates 1μg tyrosine mL/min from casein [49].

### Polyacrylamide gel electrophoresis (PAGE)

Proteins were resolved on the 12.5% continuous gel system [49]. The Tris-glycine buffer system at pH 8.8 was used to determine purity and molecular weight. The predetermined molecular weight markers of 44.3 KDa, 66.4 KDa, 97.2KDa, 116 KDa, and 200 KDa protein mixtures were loaded in the marker lane while the purified proteins were added to the gel in different wells. In individual wells, the uniduced and induced Ni-NTA purified protein was loaded along with crude protein from *E*.*coli* without insert. The gel was allowed to run in Tris-glycine buffer at 30 mA constant current for 2.5 h. After electrophoresis, the gel was stained with Coomassie Brilliant Blue R-250, and the molecular weight of the separated proteins was determined by comparing them with molecular weight standards.

## Characterization of the purified proteins

### Effect of pH and temperature on enzyme activity

The effect of pH on protease, chitinase, and fusion protein activities was recorded in various buffers of varying pH in the range of 5.0–9.0. The buffers used were sodium acetate buffer (pH 5.0 and 6.0), phosphate buffer (pH 7.0), and Tris–HCl buffer (pH 8.0 and 9.0). The 70 μL purified proteins were separately incubated in the respective buffers at 30°C for 30 min, and the pH stability and residual enzyme activities were measured as described earlier.

The effect of temperature on the activity of purified proteins was measured at different temperatures in the range from 20°C to 50°C. The purified proteins were separately incubated in phosphate buffer (pH 7) at various temperatures for 30 min, and the thermal stability and residual enzyme activities were measured as described earlier.

#### Effect of metal ions, detergent, and organic solvent on enzyme activity

The effect of metal ions on enzyme activity was analyzed using varying concentrations (1 to 100 mM) of metal ions like Co^2+^, Zn^2+^, Ca^2+^, Mg^2+^, Na^2+^, Cu^2+^, and Fe^2+^. The respective concentrations of these metal ions were separately added into each reaction mixture, followed by the addition of the purified protein 70 μL/enzyme. The stability and activities of these enzymes were measured as described earlier.

Enzyme activities were measured as described earlier. The effects of various detergents (β-Mercaptoethanol, Ethylene diamine tetra acetic acid, Sodium dodecyl sulfate, Tween 20) and organic solvents (glycerol, acetone, ethanol, methanol, butanol, and isopropanol) on the stability and activities of purified enzymes was studied by separately adding two concentration (1% and 5%) of these detergents and solvents into the reaction mixture followed by adding 70 μL purified protein [50, 51]. The enzyme activities in the absence of metal ions, detergents, and solvents were considered 100%. The percentage relative activity of enzymes was measured by dividing chemical influenced activity by enzyme activity without adding chemicals [51].

## Statistical analysis

All the experiments were carried out in five replicates, and the average of five replicates was analyzed using the Student’s t-test, and the values of p≤0.05 were considered statistically significant using SPSS Statistics for Windows, version x. 0 (SPSS Inc., Chicago, Ill., USA) [52].

## Results

### Vector construction for fusion gene with the linker

The molecular size of an amplified fragment of protease and chitinase, as evident from agarose gel electrophoresis (Fig 2A and 2B), was 1.3 kb and 1.2 kb, respectively. The comparison of fragment size and gene sequences was done with their respective sequences in the database, which confirmed the molecular weight and the size of gene sequences. The regulatory sequence of 300 bases and the *BamH1* restriction site at 5’end was ligated with individual genes. The overlapping PCR containing (G4S) 2linker was used to get a single polynucleotide sequence with a bicistron of 2.9 Kb (Fig 2B). The bicistron (Fused gene product) and monocistron (Single gene) were treated with BamH1 and KpnI to get sequences ready for ligation into the vector. The vector pUC18- Tn7 mini was double digested with BamHI and KpnI (Fig 2C) and incubated with individual genes and fusion product for the ligation. The orientation and accuracy of ligation were confirmed by restriction digestion with respective enzymes (Fig 2C).

**Fig 2:** (A) Agarose gel electrophoresis of protease and chitinase gene amplicon. Lane 1 corresponds to ladder, and Lane 2 and 4 indicate the presence of the protease gene (1.3 kb) and chitinase gene (1.2 kb), respectively; (B) Lane 1 represents DNA ladder, lane 2 to 5 represents overlapping PCR product of 2.9 kb; (C) The pUC18miniTn7FusionX Clone confirmation, Lane1- ladder, Lane 2- Unknown, Lane 3- pUC18miniTn7FusionX linearised for cloning, Lane 4- pUC18 MiniTn7 FusionX digested with BamHI and KpnI showing the insert release of 2.9 kb.

### Estimation of enzyme activities of different constructs

The zone of hydrolysis of casein was observed on the azocasien agar plate around the bacterial colonies (Fig 3A) and while the addition of 0.1% congo red on the chitin agar plate showed the zone of hydrolysis of chitin (Fig 3B).

**Fig 3:** (A and B) Activity assay of recombinant bacteria having different constructs. A = PRI—Protease, FP- Protease activity in the fusion construct. B = CHI-chitinase, FCH-chitinase activity in fusion construct.

### Protein gel electrophoresis

The recombinant fusion protein on native PAGE revealed 92 KDa, distinct protein bands, suggesting that the enzyme is a monomer and intact (Fig 4). The fusion protein was mixed with the control protein of known molecular weight, and in both lanes, it showed the band’s presence at the same place. The unknown protein was added with the protein of interest to confirm protein stability.

**Fig 4:** Native PAGE of fusion proteins expressed by *E*.*coli*. Lane 1- Protein marker (44.3 KDa, 66.4 KDa, 97.2KDa, 116 KDa, and 200 KDa), Lane 2- Sample purified using Ni-NTA column without IPTG induction; Lane 3-Sample purified using Ni-NTA column with IPTG induction; Lane 4- Crude protein without insert. Proteins were resolved on the 12.5% PAGE with standard molecular weight markers. The gel was allowed to run in Tris-glycine buffer at 30 mA constant current for 2.5 h followed by staining with Coomassie Brilliant Blue R-250. The molecular weight of the separated proteins was determined by comparing them with molecular weight standards.

### Expression and purification of proteins

Estimation of crude chitinase activity and protease activity of the recombinant expressing fusion protein revealed 1.05 folds and 1.27 folds (Table 2) increase over the individual constructs of these enzymes. Ni-NTA purified protein in the recombinant expressing fusion protein exhibited a 1.60 fold and 6.87 fold increases in the activities of chitinase and protease, respectively.

**Table 2:** The activity of recombinant proteins expressed in *E*.*coli*.

Enzyme	Stage	Unit (μM/mL/min)	Total volume (mL)	Total activity (Unit/mL)	Specific activity (Unit/mg)	Fold purification
Protease Construct	Crude	2.53	100	253.1	14.71	1.0
	Ni-NTA column	3.58	15	53.7	13.87	0.94
Protease of fusion Construct	Crude	3.21	100	321.4	18.69	1.0
	Ni-NTA column	5.72	15	85.8	22.17	1.18
Chitinase Construct	Crude	0.03	100	2.9	0.17	1.0
	Ni-NTA column	0.16	15	2.4	0.62	3.68
Chitinase of fusion Construct	Crude	0.03	100	3.1	0.18	1.0
	Ni-NTA column	1.10	15	1.5	0.38	2.11

### Characterization of purified protein

#### The effect of pH and temperature on enzyme activity

The activities of recombinant proteins were stable at different pH in a different buffer. The purified fusion protein’s optimal chitinase and protease activities were observed at pH 5.0 and 8.0, respectively (Fig 5A). Whereas the optimum temperature for the activity of purified fusion protein was found to be 30°C for both the enzyme of fusion proteins (Fig 5B). The pH and temperature optima of the fusion protein were similar to the individual proteins.

**Fig 5:** Activities of the purified proteins at pH 5–9 Values are the average of five replicates and significant at P<0.05 (A); Activities of the purified proteins at 20–50°C. Values are the average of five replicates and significant at P<0.05 (B).

#### Effect of metal ions, detergents, and organic solvents on enzyme activity

The presence of Na^2+^, Ca^2+^ and Cu^2+^ at 5 mM, and 10 mM concentrations significantly enhanced the protease activity. Metal ions such as Fe^2+^, Mg^2+^, and Zn^2+^ also improved the enzyme activities (Fig 6A). However, Na^2+^ at 5mM concentration showed enhanced chitinase activity compared to the other cations (Fig 6B). The presence of organic solvents drastically affected chitinase and protease activity in the purified fusion protein. The concentration of 1% acetone and butanol caused 40% inhibition in chitinase activity. A higher concentration (5%) of acetone drastically affected the activities of both enzymes (Fig 6C). Thus, the organic solvents showed negative impacts on the activities of both the enzyme. The purified chitinase retained 80% activity and 65% activity from its uninoculated control at 1% SDS and 5% SDS. There was a noticeable reduction in the activity of protease at both concentrations of EDTA. The addition of 2-mercaptoethanol, Tween 20 and EDTA (1%) caused a more than 50% reduction in the activity of both enzymes (Fig 6D).

**Fig 6:** The effect of various metal ions (5–10 mM) on the activity of the protease and chitinase. Values are the average of five replicates and significant at P<0.05 (A). The effect of various metal ions (5 mM and 10 mM) on the activity of chitinase. (B). Effect of denaturing agents and organic solvents at 1% and 5% on protease activity C). Effect of denaturing agents and organic solvents (1% and 5% of each) on chitinase activity (D).

## Discussion

The fragment size and gene sequences of an amplified fragment of protease and chitinase with their respective sequences in the database confirmed the molecular weight and the size of gene sequences. The map is showing the transcription termination signal, fusion gene construct and ampicillin resistant gene. The regulatory sequence of 300 bases and the *BamH1* restriction site at 5’end was ligated with individual genes. The formation of the fusion product indicated the successful ligation of individual chitinase and protease genes to form a fusion protein. The gel band of 2.9 kb size further confirmed the presence of the fusion gene sequence in the correct orientation. Growth of transformant *E*. *coli* BL21 (DE3) on chitin and casein agar plates indicated that three constructs were successfully transformed into it. Formation of the zone of hydrolysis of casein on azocasien agar plate and chitin on chitin agar plate surrounding the transformant E.coli indicated the successful expressions of chitinase and protease. The over expression of recombinant protein under IPTG induction at low temperature increases stability and solubility. Incubation period between 48–72 h yields maximum protein. The 48 h incubated samples achieved sufficient microbial concentration and low concentration of IPTG for longer time will gives better protein yield. This will lead to proper folded and biologically active protein production with least inclusion bodies formation.

The presence of fusion protein of 92 kDa on native PAGE suggested that the bifunctional enzyme is a monomer and intact. The present study results agree with the molecular weight of 44.4 KDa for *SmChiD* chitinase reported in *Serratia marcescens* [53] and 46 kDa for alkaline protease reported in *Bacillus circulans* [27]. Thus, the PAGE analysis confirms the respective size protein expressed. Mixing the fusion protein with control protein of known molecular weight followed by electrophoresis showed the band’s presence at the same place, i.e., 92 kDa indicated that a product with higher molecular weight could be efficiently expressed without any change in its activity. Sometimes, heterogonous expression of higher molecular weight proteins leads to truncated protein expression. Protein with lower molecular mass increases the stability during the post-translation stage. Various bacterial chitinase from a wide range of bacteria is possessed lower molecular mass [3, 7, 13]. The purified chitinase of *B*. *licheniformis* and *S*. *maltophila* have been reported to have molecular weights 71 kDa and 70.5 kDa, respectively [54, 55].

Increased activities of chitinase (1.60 fold) and protease (1.10 fold) in the recombinant *E*. *coli* BL21 (DE3) expressing fusion protein indicated improved activities of both enzymes in fusion construct showed enhanced activity towards the substrate. No confirmation changes occurred during the fusion of the individual proteins [56]. The thick outer membrane and limited secretion signals restrict the expression of heterogonous proteins in *E*.*coli*. However, the ompA signal sequence was successfully employed in the present study to target protein to the extracellular site. ompA sequence has been efficiently utilized to secretion exoglucanase of *C*. *fimi* from *E*. *coli* [57]. Improved enzyme activities following the cloning of genes have been reported by several scientists [58, 59]. The *SmChiD* can break down colloidal chitin in a time-dependent manner with a very low rate and produce DP2 as a significant end product [53, 58]. The chitinase used in the present study belongs to the endo acting class; it generated both reducing and non-reducing ends. The chitinase-C and N-acetyl hexosaminidase of *S*. *coelicolor* has been reported to give 90% pure GlcNAc from crab shell chitin after 8 h incubation [59]. The ChiA, ChiB, and ChiC of *S*. *marcescens* act synergistically to break chitin proficiently and give GlcNAc a major product [58, 60]. The Chi D used in the present study of *S*. *marcescens* is, an endo enzyme that produces non-reducing and reducing ends. The complete lysis of insoluble chitin requires the activity of multiple enzymes and a longer incubation time to get GlcNAc [59]. The present study reports 1 h incubation period for complete degradation of chitin into GlcNAc vis-à-vis 4 h incubation reported earlier. However, a longer incubation time will serve the purpose of breakdown complex chitin into its monomers.

The stability of activities of recombinant proteins over the range of pH and temperature optima indicated that chitinase and protease activity of fusion protein is more stable, remain more active, and retain the activities over the range of pH and temperature as compared to their counterparts [27, 53]. Other scientists have reported similar pH optima of recombinant chitinase for PbChi70 of *Paenibacillus barengoltzii* and *M*. *timonae*, respectively [13, 61]. The mesophilic temperature optima for protease and chitinase may be due to the mesophilic nature of the producing organisms. The results are in agreement with the work reported for chitinase of *Stenotrophomonas maltophilia* [55], *Bacillus licheniformis* N1 [62], and *Thermoanaerobacter tengcongensis* [63]. The serine alkaline protease Alp from *Acinetobacter* sp. IHB B 5011 (MN12) was cloned and expressed in *E*. *coli* BL21 (DE3) using the N-terminal signal sequence [25]. Similarly, a serine protease from *Bacillus* sp.WRD-2 was cloned and expressed into *E*.*coli* [64].

Improved enzyme activities in the presence of Na^2+^, Ca^2+^ and Cu^2+^, and Zn^2+^ are due to the requirement of metal ions for optimum enzyme activities. Enhanced activities protease and chitinase in the presence of Ca^2+^ ions indicated the requirement of this metal ion for the activities of these enzymes as EDTA chelate divalent cations. Similar observations have been reported in alkaliphilic *Bacillus pumilus* MCAS8 [65] and *Caldicoprobacter guelmensis* [66]. The inhibition of enzyme activities in the presence of solvents and chemicals is due to the denaturation of proteins by these solvents and chemicals. An et al. [64] reported inhibition of intracellular serine protease of *Bacillus* sp. WRD-2 in the presence of organic solvents. The inhibitory effect of organic solvents on recombinant alkaline protease and subtilisin was observed by scientists [67, 68]. Similarly, a reduction in alkaline protease activity from *Bacillus cereus* in the presence of isopropanol, methanol, ethanol, and butanol was reported [69].

The glycine-serine linker is flexible and helps in the proper folding of the enzymes. The fusion of three catalytic domains with a (G4S) 3 flexible linker showed trifunctional cellulase activity in *Saccharomyces cerevisiae* [43]. They found the higher activity of fusion protein as compared to individual clones. There was a successful fusion of *B*. *subtilis* expansin EXLX1 and *Clostridium thermocellum* endoglucanase CelD genes with a linker of different lengths and observed the highest enzyme activities in the fusion protein [70]. The fusion of two enzymes brings the active site together, and the product of one enzyme-catalyzed reaction will be immediately utilized as a substrate for the other. These strategies will be helpful for the biotransformation of various raw materials by generating a fusion of enzymes from different pathways. In the present studies, an active bifunctional protein was constructed, which presented the activities of chitinase and protease, respectively, through specific substrate analysis. E.coli has been the host of choice for cloning and heterologous expression of a wide range of proteins. Due to its well-studied genetics, faster growth rate, ability to grow on cost-effective media, safety, ample availability of vectors, ease in extracellular production using signal sequences, and convenient in the extraction of the product, E.coli is preferred over the other hosts. The fusion and Co-expression of endoglucanase and beta-glucosidase were successfully carried out in *E*.*coli* [36]. Several other reports indicating fusion and co-expression of proteins belong to endoglucanase and β-glucosidase for hydrolyzing sugarcane bagasse [38]. Thus chitinase and protease can be successfully fused and expressed in *E*.*coli* without changing their catalytic activities, properties, and kinetics. However, more studies on kinetics, molecular aspects, and protein characterization are required to claim the success of fusion protein.

## Conclusion

Heterologous expression of the fusion protein is successfully carried out by using a pUC18-T7 mini vector with *an ompA* signal sequence. The bicistronic vector expresses fusion protein using glycine-serine linker as a single peptide appears to be a feasible and cost-effective approach of combining two enzymes in a single protein. A single fusion protein exhibiting the activities of two enzymes can effectively degrade the complex substrates made up of chitin and protein. Improved activities of these enzymes in fusion protein offer higher biodegradation rates than the biodegradation by a single enzyme. Moreover, the biodegradation of chitin mediated by fusion protein holds merits in terms of safety, higher productivity, and the formation of a good number of monomers. Cloning of genes of two enzymes in the fast-growing host that also gives better co-expression, higher enzyme yield, and improved activities compared to individual enzymes will have more and broader applications. This report is the first report on a single fusion protein that has chitinase and protease activities. However, further studies on enzyme kinetics, molecular studies on genes involved, and studies on protein structure may further enhance the activities, yield, and stability of fusion under diverse physicochemical conditions.

## Supporting information

S1 Fig (JPG)

S2 Fig (JPG)

S3 Fig (JPG)

S4 Fig (JPG)

S1 Raw images (PDF)
